# A Computational Approach for the Calculation of Temperature Distribution in Casting-Mould Heterogeneous System with Fractional Order

**DOI:** 10.1155/2022/3648277

**Published:** 2022-07-26

**Authors:** Xiankang Luo, Muhammad Nadeem, Muhammad Imran Asjad, Mohammed S. Abdo

**Affiliations:** ^1^Faculty of Science, Yibin University, Yibin 644000, China; ^2^Department of Mathematics, University of Management and Technology, Lahore 54770, Pakistan; ^3^Department of Mathematics, Hodeidah University, Al-Hudaydah, Yemen

## Abstract

The purpose of this paper is to investigate the approximate solution of the casting-mould heterogeneous system with Caputo derivative under the homotopy idea. The symmetry design of the system contains the integer partial differential equations and the fractional-order partial differential equations. We apply Yang transform homotopy perturbation method (*𝒴*T-HPM) to find the approximate solution of temperature distribution in the casting-mould heterogeneous system. The *𝒴*T-HPM is a combined form of Yang transform (*𝒴*T) and the homotopy perturbation method (HPM) using He's polynomials. Some examples are provided to demonstrate the superiority of the suggested technique. The significant findings reveal that *𝒴*T-HPM minimizes the enormous without imposing any assumptions. Due to its powerful and robust support for nonlinear problems, this approach presents a remarkable appearance in the functional studies of fractal calculus.

## 1. Introduction

A differential problem of symmetry is a modification that generates the differential equation continuously in such a way that these symmetries can help to achieve the solution of the differential equation. Solving these equations is sometimes easier than solving the original differential equations. In the past few decades, nonlinear fractional differential equations (FDEs) in mathematical physics have been contending for a prominent role in a variety of fields, including biological research, applied science, signal processing, control theory, finance, and fractal dynamics [1–3]. Debnath [4] presents some recent applications of fractional calculus and obtained the numerical computation of fractional derivatives and integrals. Heydari et al. [5] applied the Legendre polynomials to obtain the numerical solution of nonlinear fractal-fractional optimal control problems. Wang and Wang [6] employed a semi-inverse method to obtain the fractal variational principles for two different types of discontinuous plasma physics. FDEs are the generalized forms of the integer-order differential equations but some nonlinear mathematical models of integer-order derivatives do not implement well in most of the circumstances [7–9]. This is because integer-order derivatives are limited operators that are unsuitable for infinite variance, whereas the fractional-order derivatives are global to account for neighborhood dominance.

Various types of differential equations with the fractional derivative can be used to precisely characterize many proceedings of physics and engineering. Khan et al. [10] constructed an operator using the Caputo fractional differentiation to validate the performance of this approach. The challenge of discovering approximate and exact solutions to FDEs is much critical. The homotopy perturbation technique (HPM) [11] is a well-known method for obtaining series solutions to a variety of linear and nonlinear differential equations of arbitrary order. Many powerful and efficient strategies have been proposed such as Laplace homotopy perturbation method [12], weighted least squares method [13], iterative method [14], homotopy perturbation Sumudu transform method [15], Elzaki transform decomposition approach [16], Laplace decomposition method [17], and natural homotopy transform method [18] with a logic sensitivity function and small diffusivity. Grzymkowski et al. [19] employed HPM whereas Tripathi and Mishra [20] adopted HPM together with the Laplace transform to determine the temperature distribution in the casting-mould heterogeneous system as a continuous function, which is particularly useful for analyzing the mould. Vanani et al. [21] used a weighted approach based on HPM to solve the heat equation in the cast-mould heterogeneous domain. Later, this proposed approach has also been examined in more than one spatial dimension, indicating that this method has a broader application in nonlinear PDE systems [22, 23]. This study is particularly powerful for fractal theory and fractal calculus, and it can be seen as dependable in getting analytical solutions and suitable for other nonlinear issues [24–26].

This study presents the idea of *𝒴*T-HPM to obtain the solution of casting-mould heterogeneous system with fractional order in Caputo sense. Yang transform coupled with the homotopy perturbation method presents the results in the form of series and this series approaches to the exact solution very rapidly. The quality of the current method is appropriate to provide the analytical results to the given examples. This study is summarized as follows: in Section 2, we start with some primary definitions in Caputo sense. In Sections 3 and 4, we formulate the problem for the implementation of *𝒴*T-HPM. In Section 6, we apply this scheme to two numerical problems to show its capability and efficiency. Results and discussion with concluding remarks are given in Sections 7 and 8.

## 2. Preliminary Concepts

In this segment, we demonstrate some fundamental properties of fractional calculus along with Yang transform, which help to construct the idea of *𝒴*T-HPM.

**Definition 1 .**

The fractional-order derivative in Caputo sense is given as [27]

(1) $$\begin{array}{c} D_{\eta }^{\alpha }\Psi \left(\theta ,\eta \right)=\frac{1}{\Gamma \left(\lambda -\alpha \right)}\int_{0}^{\eta }\;{\left(\eta -\rho \right)}^{\lambda -\alpha -1}\Psi \left(\varphi ,\rho \right)d\rho ,\lambda -1<\alpha \leq \lambda ,\;\lambda \in \mathbb{N}. \end{array}$$

**Definition 2 .**

Recently, Yang [28] introduced the Yang-Laplace transform that if Ψ(*η*) is a function, then *𝒴*T can be written as

(2) $$\begin{array}{c} Y\left[\Psi \left(\eta \right)\right]=M\left(w\right)=\int_{0}^{\infty }\;e^{-\left(\eta /w\right)}\Psi \left(\eta \right)d\eta ,\eta ,w>0. \end{array}$$

**Definition 3 .**

The inverse transform *𝒴*^−1^ is defined as

(3) $$\begin{array}{c} Y^{-1}\left[M\left(w\right)\right]=\Psi \left(\eta \right)\text{red}, \end{array}$$

where *𝒴*^−1^ is the inverse Yang operator.

**Definition 4 .**

The Yang transform for *n*th derivatives is defined a [28]

(4) $$\begin{array}{c} Y\left[\Psi^{n}\left(\eta \right)\right]=\frac{M\left(w\right)}{w^{n}}-\overset{n-1}{\underset{\lambda =0}{\sum }}\;\frac{\Psi^{\lambda }\left(0\right)}{w^{n-\lambda -1}},\;n=1,2,3,\cdots . \end{array}$$

**Definition 5 .**

The Yang transform for fractional-order derivatives is defined as [29]

(5) $$\begin{array}{c} Y\left[\Psi^{\alpha }\left(\eta \right)\right]=\frac{M\left(w\right)}{w^{\alpha }}-\overset{n-1}{\underset{\lambda =0}{\sum }}\;\frac{\Psi^{\lambda }\left(0\right)}{w^{\alpha -\lambda -1}},\;0<\alpha \leq n. \end{array}$$

## 3. Remarks

The *𝒴*T of some helpful expressions are as follows:

(6) $$\begin{array}{c} Y\left[1\right]=w,\\ Y\left[\eta \right]=w^{2},\\ Y\left[\eta^{\lambda }\right]=\Gamma \left(\lambda +1\right)w^{\lambda +1}. \end{array}$$

## 4. The Description of the Problem

In this segment, we formulate the casting-mould system to analyze the temperature distribution. Let us consider, two regions, Ψ(*θ*, *η*) indicating for casting and *Φ*(*θ*, *η*) for mould on the boundary of the problem as shown in Figure 1, such that

(7) $$\begin{array}{c} \begin{array}{cc} \Psi =\left(\theta ,\eta \right)\text{: }\theta \in \left[\theta_{1},0\right], & \eta \in \left[0,\eta^{*}\right),\\ \Phi =\left(\theta ,\eta \right)\text{: }\theta \in \left[0,\theta_{2}\right], & \eta \in \left[0,\eta^{*}\right), \end{array} \end{array}$$

with the boundaries on these domains *δ*_*i*_,  *i* = 1, 2, 3, 4, 5 are distributed as

(8) $$\begin{array}{c} \begin{array}{c} \delta_{1}=\left\{\left(\theta ,0\right)\text{: }\theta \in \left(\theta_{1},0\right)\right\},\\ \delta_{2}=\left\{\left(0,\eta \right)\text{: }\theta \in \left[0,\eta^{*}\right]\right\},\\ \delta_{3}=\left\{\left(\theta_{1},\eta \right)\text{: }\theta \in \left[0,\eta^{*}\right]\right\},\\ \delta_{4}=\left\{\left(\theta ,0\right)\text{: }\theta \in \left[0,\theta_{2}\right]\right\},\\ \delta_{5}=\left\{\left(\theta_{2},\eta \right)\text{: }\theta \in \left[0,\eta^{*}\right]\right\}. \end{array} \end{array}$$

These functions satisfy the heat conduction equation inside the domains such as:

(9) $$\begin{array}{c} \begin{array}{c} \frac{\partial^{\alpha }\Psi \left(\theta ,\eta \right)}{\partial \eta^{\alpha }}=a\frac{\partial^{2}\Psi \left(\theta ,\eta \right)}{\partial \theta^{2}},\left(\theta ,\eta \right)\in \Psi ,\\ \frac{\partial^{\alpha }\Phi \left(\theta ,\eta \right)}{\partial \eta^{\alpha }}=b\frac{\partial^{2}\Phi \left(\theta ,\eta \right)}{\partial \theta^{2}},\;\left(\theta ,\eta \right)\in \Phi , \end{array} \end{array}$$

where *∂*^*α*^/*∂η*^*α*^ is the derivative of functions *Φ*(*θ*, *η*) and Ψ(*θ*, *η*) order *α* in Caputo sense, *a* and *b* are the thermal diffusivity, Ψ and *Φ* represent the temperature, and *η* and *θ* refer to the time and spatial, respectively [30]. These boundaries satisfy the following initial and boundary conditions:

(10) $$\begin{array}{c} \begin{array}{c} \Psi \left(\theta ,0\right)=\phi_{1}\left(\theta \right),\;\text{on }\delta_{1},\\ \Phi \left(\theta ,0\right)=\phi_{2}\left(\theta \right),\;\text{on }\delta_{4},\\ \begin{array}{c} \Psi \left(\theta_{1},\eta \right)=\psi \left(\eta \right),\;\text{on }\delta_{3},\\ \frac{\partial \Phi \left(\theta_{2},\eta \right)}{\partial \theta }=q\left(\eta \right),\;\text{on }\delta_{5},\\ \begin{array}{c} \Psi \left(0,\eta \right)=\Phi \left(0,\eta \right),\;\text{on }\delta_{2},\\ \zeta_{1}\frac{\partial \Psi \left(0,\eta \right)}{\partial \theta }=\zeta_{2}\frac{\Phi \left(0,\eta \right)}{\partial \theta },\;\text{on }\delta_{2}. \end{array} \end{array} \end{array} \end{array}$$

The selection of these boundary conditions is an important task for the determination of the casting-mould problem.

## 5. Idea of *𝒴*T-HPM

In this part, we will demonstrate the concept of YHPTM. Let us assume fractional-order PDE such as

(11) $$\begin{array}{c} D_{\eta }^{\alpha }\Psi \left(\theta ,\eta \right)+R\Psi \left(\theta ,\eta \right)+N\Psi \left(\theta ,\eta \right)=g\left(\theta ,\eta \right), \end{array}$$

(12) $$\begin{array}{c} \Psi \left(\theta ,0\right)=h\left(\theta \right), \end{array}$$

where *R* and *N* are linear and nonlinear differential operators, respectively, and *g*(*θ*, *η*) is called the source function. Applying the *𝒴*T to Equation (11),

(13) $$\begin{array}{c} \frac{1}{w^{\alpha }}Y\left[\Psi \left(\theta ,\eta \right)-w\Psi \left(\theta ,0\right)\right]=-Y\left[R\left(\Psi \left(\theta ,\eta \right)\right)+N\left(\Psi \left(\theta ,\eta \right)\right)+Y\left[g\left(\theta ,\eta \right)\right]\right],\\ Y\left[\Psi \left(\theta ,\eta \right)\right]=wh\left(\theta \right)-w^{\alpha }\left[Y\left[R\left(\Psi \left(\theta ,\eta \right)\right)+N\left(\Psi \left(\theta ,\eta \right)\right)\right]\right]+Y\left[g\left(\theta ,\eta \right)\right]. \end{array}$$

By using inverse *𝒴*,

(14) $$\begin{array}{c} \Psi \left(\theta ,\eta \right)=\Psi \left(\theta ,0\right)-Y^{-1}\left[w^{\alpha }\left[Y\left[R\left(\Psi \left(\theta ,\eta \right)\right)+N\left(\Psi \left(\theta ,\eta \right)\right)\right]\right]+Y\left[g\left(\theta ,\eta \right)\right]\right]. \end{array}$$

However, HPM is stated as

(15) $$\begin{array}{c} \Psi \left(\theta ,\eta \right)=\overset{\infty }{\underset{i=0}{\sum }}\;p^{i}\Psi_{i}\left(\theta ,\eta \right), \end{array}$$

where *p* is the homotopy parameter and

(16) $$\begin{array}{c} N\Psi \left(\theta ,\eta \right)=\overset{\infty }{\underset{i=0}{\sum }}\;p^{i}H_{i}\Psi \left(\theta ,\eta \right). \end{array}$$

The following strategy can be operated to acquire He's polynomials:

(17) $$\begin{array}{c} H_{i}\left(\Psi_{0}+\Psi_{1}+\cdots +\Psi_{i}\right)=\frac{1}{n!}\frac{\partial^{i}}{\partial p^{i}}{\left(N\left(\overset{\infty }{\underset{i=0}{\sum }}\;p^{i}\Psi_{i}\right)\right)}_{p=0},\;n=0,1,2,\cdots . \end{array}$$

With the help of Equations (15) and (16), we can get Equation (14) such as

(18) $$\begin{array}{c} \overset{\infty }{\underset{i=0}{\sum }}\;p^{i}\Psi_{i}\left(\theta ,\eta \right)=\Psi \left(\theta ,0\right)-pY^{-1}\left[w^{\alpha }Y\left\{R\left(\overset{\infty }{\underset{i=0}{\sum }}\;p^{i}\Psi_{i}\left(\theta ,\eta \right)\right)+\overset{\infty }{\underset{i=0}{\sum }}\;p^{i}H_{n}\Psi_{i}\left(\theta ,\eta \right)\right\}\right]. \end{array}$$

We can get the following terms by evaluating the *p* components

(19) p^0:Ψ0θ,η=Ψθ,0,p1:Ψ1θ,η=−Y−1wαYRΨ0θ,η+H0Ψ,p2:Ψ2θ,η=−Y−1wαYRΨ1θ,η+H1Ψ,p3:Ψ3θ,η=−Y−1wαYRΨ2θ,η+H2Ψ,⋮pi:Ψiθ,η=−Y−1wαYRΨiθ,η+HiΨ.

Thus, we can summarize the set of Equation (19) in the series form such as

(20) $$\begin{array}{c} \Psi \left(\theta ,\eta \right)=\Psi_{0}\left(\theta ,\eta \right)+\Psi_{1}\left(\theta ,\eta \right)+\Psi_{2}\left(\theta ,\eta \right)+\cdots ,\\ \Psi \left(\theta ,\eta \right)=\underset{N⟶\infty }{\lim}\overset{N}{\underset{n=0}{\sum }}\;\Psi_{n}\left(\theta ,\eta \right). \end{array}$$

## 6. Numerical Examples

Case I: let us consider

(21) $$\begin{array}{c} \begin{array}{c} \theta_{1}=-1,\;\theta_{2}=1\;a=\frac{1}{4},\;b=1,\\ \zeta_{1}=1,\;\zeta_{2}=2,\;\Psi_{0}\left(\theta ,\eta \right)=e^{2\theta },\;\Phi_{0}\left(\theta ,\eta \right)=e^{\theta }. \end{array} \end{array}$$

Thus, system of Equation (9) becomes

(22) $$\begin{array}{c} \begin{array}{c} \frac{\partial^{\alpha }\Psi }{\partial \eta^{\alpha }}=\frac{1}{4}\frac{\partial^{2}\Psi }{\partial \theta^{2}},\\ \frac{\partial^{\alpha }\Phi }{\partial \eta^{\alpha }}=\frac{\partial^{2}\Phi }{\partial \theta^{2}}. \end{array} \end{array}$$

Now, taking *𝒴*T and using its property definition, we get

(23) $$\begin{array}{c} Y\left[\Psi \left(\theta ,\eta \right)\right]=w\Psi \left(\theta ,0\right)+w^{\alpha }Y\left[\frac{1}{4}\frac{\partial^{2}\Psi }{\partial \theta^{2}}\right],\\ Y\left[\Phi \left(\theta ,\eta \right)\right]=w\Phi \left(\theta ,0\right)+w^{\alpha }Y\left[\frac{\partial^{2}\Phi }{\partial \theta^{2}}\right]. \end{array}$$

Thus, inverse *𝒴*T takes place as

(24) $$\begin{array}{c} \begin{array}{c} \Psi \left(\theta ,\eta \right)=\Psi \left(\theta ,0\right)+Y^{-1}\left[w^{\alpha }Y\left\{\frac{1}{4}\frac{\partial^{2}\Psi }{\partial \theta^{2}}\right\}\right],\\ \Phi \left(\theta ,\eta \right)=\Phi \left(\theta ,0\right)+Y^{-1}\left[w^{\alpha }Y\left\{\frac{\partial^{2}\Phi }{\partial \theta^{2}}\right\}\right]. \end{array} \end{array}$$

Using the initial condition Equation (21) into Equation (24), we get

(25) $$\begin{array}{c} \Psi \left(\theta ,\eta \right)=e^{2\theta }+Y^{-1}\left[w^{\alpha }Y\left\{\frac{1}{4}\frac{\partial^{2}\Psi }{\partial \theta^{2}}\right\}\right],\\ \Phi \left(\theta ,\eta \right)=e^{\theta }+Y^{-1}\left[w^{\alpha }Y\left\{\frac{\partial^{2}\Phi }{\partial \theta^{2}}\right\}\right]. \end{array}$$

Applying HPM to get with He's polynomials, we get

(26) $$\begin{array}{c} \begin{array}{c} \overset{\infty }{\underset{i=0}{\sum }}\;p^{i}\Psi_{i}\left(\theta ,\eta \right)=e^{2\theta }+Y^{-1}\left[w^{\alpha }Y\left(\frac{1}{4}\overset{\infty }{\underset{i=0}{\sum }}\;p^{i}\frac{\partial^{2}\Psi_{i}}{\partial \theta^{2}}\right)\right],\\ \overset{\infty }{\underset{i=0}{\sum }}\;p^{i}\Phi_{i}\left(\theta ,\eta \right)=e^{\theta }+Y^{-1}\left[w^{\alpha }Y\left(\overset{\infty }{\underset{i=0}{\sum }}\;p^{i}\frac{\partial^{2}\Phi_{i}}{\partial \theta^{2}}\right)\right]. \end{array} \end{array}$$

Start with the initial condition to get the following iteration in the form of series

(27) $$\begin{array}{c} \Psi_{0}\left(\theta ,\eta \right)=\Psi \left(\theta ,0\right)=e^{2\theta },\\ \Phi_{0}\left(\theta ,\eta \right)=\Phi \left(\theta ,0\right)=e^{\theta },\\ \Psi_{1}\left(\theta ,\eta \right)=Y^{-1}\left[w^{\alpha }Y\left(\frac{1}{4}\frac{\partial^{2}\Psi_{0}}{\partial \theta^{2}}\right)\right]=e^{2\theta }\frac{\eta^{\alpha }}{\Gamma \left(1+\alpha \right)},\\ \Phi_{1}\left(\theta ,\eta \right)=Y^{-1}\left[w^{\alpha }Y\left(\frac{\partial^{2}\Phi_{0}}{\partial \theta^{2}}\right)\right]=e^{\theta }\frac{\eta^{\alpha }}{\Gamma \left(1+\alpha \right)},\\ \Psi_{2}\left(\theta ,\eta \right)=Y^{-1}\left[w^{\alpha }Y\left(\frac{1}{4}\frac{\partial^{2}\Psi_{1}}{\partial \theta^{2}}\right)\right]=e^{2\theta }\frac{\eta^{2\alpha }}{\Gamma \left(1+2\alpha \right)},\\ \Phi_{2}\left(\theta ,\eta \right)=Y^{-1}\left[w^{\alpha }Y\left(\frac{\partial^{2}\Phi_{1}}{\partial \theta^{2}}\right)\right]=e^{\theta }\frac{\eta^{2\alpha }}{\Gamma \left(1+2\alpha \right)},\\ \Psi_{3}\left(\theta ,\eta \right)=Y^{-1}\left[w^{\alpha }Y\left(\frac{1}{4}\frac{\partial^{2}\Psi_{2}}{\partial \theta^{2}}\right)\right]=e^{2\theta }\frac{\eta^{3\alpha }}{\Gamma \left(1+3\alpha \right)},\\ \Phi_{3}\left(\theta ,\eta \right)=Y^{-1}\left[w^{\alpha }Y\left(\frac{\partial^{2}\Phi_{2}}{\partial \theta^{2}}\right)\right]=e^{\theta }\frac{\eta^{3\alpha }}{\Gamma \left(1+3\alpha \right)},\\ \vdots \end{array}$$

Consequently, the series may be demonstrated as:

(28) $$\begin{array}{c} \Psi \left(\theta ,\eta \right)=\Psi_{0}+\Psi_{1}+\Psi_{2}+\Psi_{3}+\cdots ,\\ \Phi \left(\theta ,\eta \right)=\Phi_{0}+\Phi_{1}+\Phi_{2}+\Phi_{3}+\cdots , \end{array}$$

which can be written as follows

(29) $$\begin{array}{c} \Psi \left(\theta ,\eta \right)=e^{2\theta }\left[1+\frac{\eta^{\alpha }}{\Gamma \left(1+\alpha \right)}+\frac{\eta^{2\alpha }}{\Gamma \left(1+2\alpha \right)}+\frac{\eta^{3\alpha }}{\Gamma \left(1+3\alpha \right)}+\cdots \right],\\ \Phi \left(\theta ,\eta \right)=e^{\theta }\left[1+\frac{\eta^{\alpha }}{\Gamma \left(1+\alpha \right)}+\frac{\eta^{2\alpha }}{\Gamma \left(1+2\alpha \right)}+\frac{\eta^{3\alpha }}{\Gamma \left(1+3\alpha \right)}+\cdots \right]. \end{array}$$

For *α* = 1, the above equations may reduce to the classical casting system

(30) $$\begin{array}{c} \Psi \left(\theta ,\eta \right)=e^{2\theta +\eta },\\ \Phi \left(\theta ,\eta \right)=e^{\theta +\eta }. \end{array}$$

Case II: let us consider again

(31) $$\begin{array}{c} \begin{array}{c} \theta_{1}=-1,\;\theta_{2}=1\;a=\frac{1}{4},\;b=1,\\ \zeta_{1}=1,\;\zeta_{2}=2,\;\Psi_{0}\left(\theta ,\eta \right)=2+e^{2\theta },\;\Phi_{0}\left(\theta ,\eta \right)=e^{\theta }. \end{array} \end{array}$$

Thus, system of Equation (9) becomes

(32) $$\begin{array}{c} \begin{array}{c} \frac{\partial^{\alpha }\Psi }{\partial \eta^{\alpha }}=\frac{1}{4}\frac{\partial^{2}\Psi }{\partial \theta^{2}},\\ \frac{\partial^{\alpha }\Phi }{\partial \eta^{\alpha }}=\frac{\partial^{2}\Phi }{\partial \theta^{2}}. \end{array} \end{array}$$

According to *𝒴*T-HPM, we get

(33) $$\begin{array}{c} \begin{array}{c} \overset{\infty }{\underset{i=0}{\sum }}\;p^{i}\Psi_{i}\left(\theta ,\eta \right)=e^{2\theta }+Y^{-1}\left[w^{\alpha }Y\left(\frac{1}{4}\overset{\infty }{\underset{i=0}{\sum }}\;p^{i}\frac{\partial^{2}\Psi_{i}}{\partial \theta^{2}}\right)\right],\\ \overset{\infty }{\underset{i=0}{\sum }}\;p^{i}\Phi_{i}\left(\theta ,\eta \right)=e^{\theta }+Y^{-1}\left[w^{\alpha }Y\left(\overset{\infty }{\underset{i=0}{\sum }}\;p^{i}\frac{\partial^{2}\Phi_{i}}{\partial \theta^{2}}\right)\right]. \end{array} \end{array}$$

Start with the initial condition to get the following iteration in the form of series

(34) $$\begin{array}{c} \Psi_{0}\left(\theta ,\eta \right)=2+e^{2\theta },\\ \Phi_{0}\left(\theta ,\eta \right)=e^{\theta },\\ \Psi_{1}\left(\theta ,\eta \right)=Y^{-1}\left[w^{\alpha }Y\left(\frac{1}{4}\frac{\partial^{2}\Psi_{0}}{\partial \theta^{2}}\right)\right]=e^{2\theta }\frac{\eta^{\alpha }}{\Gamma \left(1+\alpha \right)},\\ \Phi_{1}\left(\theta ,\eta \right)=Y^{-1}\left[w^{\alpha }Y\left(\frac{\partial^{2}\Phi_{0}}{\partial \theta^{2}}\right)\right]=e^{\theta }\frac{\eta^{\alpha }}{\Gamma \left(1+\alpha \right)},\\ \Psi_{2}\left(\theta ,\eta \right)=Y^{-1}\left[w^{\alpha }Y\left(\frac{1}{4}\frac{\partial^{2}\Psi_{1}}{\partial \theta^{2}}\right)\right]=e^{2\theta }\frac{\eta^{2\alpha }}{\Gamma \left(1+2\alpha \right)},\\ \Phi_{2}\left(\theta ,\eta \right)=Y^{-1}\left[w^{\alpha }Y\left(\frac{\partial^{2}\Phi_{1}}{\partial \theta^{2}}\right)\right]=e^{\theta }\frac{\eta^{2\alpha }}{\Gamma \left(1+2\alpha \right)},\\ \Psi_{3}\left(\theta ,\eta *\right)=Y^{-1}\left[w^{\alpha }Y\left(\frac{1}{4}\frac{\partial^{2}\Psi_{2}}{\partial \theta^{2}}\right)\right]=e^{2\theta }\frac{\eta^{3\alpha }}{\Gamma \left(1+3\alpha \right)},\\ \Phi_{3}\left(\theta ,\eta \right)=Y^{-1}\left[w^{\alpha }Y\left(\frac{\partial^{2}\Phi_{2}}{\partial \theta^{2}}\right)\right]=e^{\theta }\frac{\eta^{3\alpha }}{\Gamma \left(1+3\alpha \right)},\\ \vdots \end{array}$$

Consequently, the series may be demonstrated as:

(35) $$\begin{array}{c} \Psi \left(\theta ,\eta \right)=\Psi_{0}+\Psi_{1}+\Psi_{2}+\Psi_{3}+\cdots ,\\ \Phi \left(\theta ,\eta \right)=\Phi_{0}+\Phi_{1}+\Phi_{2}+\Phi_{3}+\cdots , \end{array}$$

which can be written as follows:

(36) $$\begin{array}{c} \Psi \left(\theta ,\eta \right)=2+e^{2\theta }\left[1+\frac{\eta^{\alpha }}{\Gamma \left(1+\alpha \right)}+\frac{\eta^{2\alpha }}{\Gamma \left(1+2\alpha \right)}+\frac{\eta^{3\alpha }}{\Gamma \left(1+3\alpha \right)}+\cdots \right],\\ \Phi \left(\theta ,\eta \right)=e^{\theta }\left[1+\frac{\eta^{\alpha }}{\Gamma \left(1+\alpha \right)}+\frac{\eta^{2\alpha }}{\Gamma \left(1+2\alpha \right)}+\frac{\eta^{3\alpha }}{\Gamma \left(1+3\alpha \right)}+\cdots \right]. \end{array}$$

For *α* = 1, the above equations may reduce to the classical casting system

(37) $$\begin{array}{c} \Psi \left(\theta ,\eta \right)=2+e^{2\theta +\eta },\\ \Phi \left(\theta ,\eta \right)=e^{\theta +\eta }. \end{array}$$

## 7. Results and Discussion

In case I, Figures 2(a)–2(d) indicate the surface solution of casting system, whereas Figures 3(a)–3(d) indicates the surface solution of mould system, respectively, with fractional order *α* = 0.25, *α* = 0.50, *α* = 0.75, and *α* = 1 at *θ* = 5 and *η* = 1. Figures 4 and 5 indicate the graphical results of Ψ(*θ*, *η*) and *Φ*(*θ*, *η*), respectively, for different values of *α* at *θ* = 1 and *η* = 0.1.  Table 1 represents the absolute error of the casting system, and Table 2 represents absolute error of the mould system.

In case II, Figures 6(a)–6(d) indicate the surface solution of casting system with fractional order *α* = 0.25, *α* = 0.50, *α* = 0.75, and *α* = 1 at *θ* = 2 and *η* = 2.  Figure 7 indicates the graphical results of Ψ(*θ*, *η*) for different values of *α* at *θ* = 2 and *η* = 0.1. However, the graphical results for the mould system remain same because only changing the initial condition in casting system is studied to show the performance of this approach in this case.  Table 3 represents the absolute error of casting system.

These graphical results reveal that they are virtually similar and validate towards the exact solutions, which encourages us to interpret the physical behavior of the coupled system. The solutions results are demonstrated in both 2D and 3D to realize the physical description of the coupled system.

## 8. Conclusion

In this survey, we successfully utilized *𝒴*T-HPM to investigate the approximate solution of the casting-mould heterogeneous system with the Gerasimov-Caputo derivative. This approach does not involve any hypothesis and restriction of variables to ruin the nature of the problems in the recurrence relation. Two examples are tested to verify the excellent performance of this hybrid scheme. It is seen that *𝒴*T-HPM has less computational effort which shows that the solution of the system of PDEs has a fast rate of convergence. We performed all the calculations with the help of Wolfram Mathematica software 11.0.1. The graphical representation of surface solution and plot distributing validate that *𝒴*T-HPM results are very precise and effective which demonstrates that this approach is very simple and straightforward for other nonlinear evolution problems with fractal derivatives in the future demands.

## Figures and Tables

**Figure 1:** Domain of the problem.

**Figure 2:** The surfaces solution of Ψ(*θ*, *η*) for distinct values of *α*.

**Figure 3:** Plot of Ψ(*θ*, *η*) for different values of *α*.

**Figure 4:** The surfaces solution of *Φ*(*θ*, *η*) for distinct values of *α*.

**Figure 5:** Plot of *Φ*(*θ*, *η*) for different values of *α*.

**Figure 6:** The surfaces solution of Ψ(*θ*, *η*) for distinct values of *α*.

**Figure 7:** Plot of Ψ(*θ*, *η*) for different values of *α*.

**Table 1:** Consider *θ* = 0.001 at *α* = 1 for casting system.

*t*	Exact solution	Approximate solution	Absolute error
.25	1.2866	1.2866	0.000
.50	1.65202	1.65202	0.000
.75	2.12124	2.12124	0.000
.0	2.72372	2.7237	0.00002
.25	3.49716	3.49733	0.00017
.50	4.49066	4.4899	0.0007
.75	5.76612	5.76342	0.0027
.0	7.40385	7.39573	0.00812

**Table 2:** Consider *θ* = 0.005 at *α* = 1 for mould system.

*t*	Exact solution	Approximate solution	Absolute error
.25	1.29046	1.29046	0.000
.50	1.65699	1.65699	0.000
.75	2.12761	2.12761	0.000
.0	2.73191	2.73188	0.0003
.25	3.50784	3.50767	0.00017
.50	4.50415	4.50339	0.00076
.75	5.78345	5.78074	0.00271
.0	7.42609	7.41795	0.00814

**Table 3:** Consider *θ* = 0.005 at *α* = 1 for casting system.

*t*	Exact solution	Approximate solution	Absolute error
.25	3.29693	3.29693	0.000
.50	3.66529	3.66529	0.000
.75	4.13828	4.13827	0.00001
.0	4.7456	4.74557	0.00003
.25	5.52542	5.52525	0.00017
.50	6.52673	6.52596	0.00077
.75	7.81244	7.80972	0.00272
.0	9.46332	9.45513	0.00819

## Data Availability

All the data are available within the article.

## References

[1] Guo S., Mei L., Li Y., Sun Y. (2012). The improved fractional sub-equation method and its applications to the space–time fractional differential equations in fluid mechanics. *Physics Letters A*.

[2] Owolabi K. M., Atangana A., Akgul A. (2020). Modelling and analysis of fractal-fractional partial differential equations: application to reaction-diffusion model. *Alexandria Engineering Journal*.

[3] Wang K. (2022). Fractal solitary wave solutions for fractal nonlinear dispersive boussinesq-like models. *Fractals*.

[4] Debnath L. (2003). Recent applications of fractional calculus to science and engineering. *International Journal of Mathematics and Mathematical Sciences*.

[5] Heydari M. H., Atangana A., Avazzadeh Z. (2021). Numerical solution of nonlinear fractal-fractional optimal control problems by legendre polynomials. *Mathematical Methods in the Applied Sciences*.

[6] Wang K.-L., Wang H. (2022). Fractal variational principles for two different types of fractal plasma models with variable coefficients. *Fractals*.

[7] Baleanu D., Machado J. A. T., Luo A. C. (2011). *Fractional Dynamics and Control*.

[8] Miller K. S., Ross B. (1993). *An Introduction to the Fractional Calculus and Fractional Differential Equations*.

[9] Tajadodi H., Khan Z. A., Gómez-Aguilar J. F., Khan A., Khan H. (2021). Exact solutions of conformable fractional differential equations. *Results in Physics*.

[10] Khan Y., Khan A., Shaeel M., Akgül A. (2021). Two dimensional Laplace transform coupled with the Marichev–Saigo–Maeda integral operator and the generalized Incomplete hypergeometric function. *Symmetry*.

[11] Wu Y., He J.-H. (2018). Homotopy perturbation method for nonlinear oscillators with coordinate dependent mass. *Results in Physics*.

[12] Morales-Delgado V. F., Gómez-Aguilar J. F., Kumar S., Taneco-Hernández M. A. (2018). Analytical solutions of the Keller-Segel chemotaxis model involving fractional operators without singular kernel. *The European Physical Journal Plus*.

[13] Lone S. A., Anwar S., Sindhu T. N., Jarad F. (2022). Some estimation methods for mixture of extreme value distributions with simulation and application in medicine. *Results in Physics*.

[14] Atangana A. (2015). Extension of the Sumudu homotopy perturbation method to an attractor for one-dimensional Keller–Segel equations. *Applied Mathematical Modelling*.

[15] Sharma D., Samra G. S., Singh P. (2020). Approximate solution for fractional attractor one-dimensional Keller-Segel equations using homotopy perturbation Sumudu transform method. *Nonlinear Engineering*.

[16] Khan H., Khan A., Kumam P., Baleanu D., Arif M. (2020). An approximate analytical solution of the Navier–Stokes equations within Caputo operator and Elzaki transform decomposition method. *Adv. Difference Equ.*.

[17] Khan Y. (2009). An Effective modification of the Laplace decomposition method for nonlinear equations. *International Journal of Nonlinear Sciences and Numerical Simulation*.

[18] Liu H., Khan H., Shah R., Alderremy A. A., Aly S., Baleanu D. (2020). On the fractional view analysis of Keller–Segel equations with sensitivity functions. *Complexity*.

[19] Grzymkowski R., Pleszczyński M., Słota D. (2009). Application of the Adomian decomposition method for solving the heat equation in the cast-mould heterogeneous domain. *Archives of Foundry Engineering*.

[20] Tripathi R., Mishra H. K. (2018). Application of homotopy perturbation method using Laplace transform intended for determining the temperature in the heterogeneous casting-mould system. *Differential Equations and Dynamical Systems*.

[21] Vanani S. K., Yildirim A., Soleymani F., Khan M., Tutkun S. (2013). Solution of the heat equation in the cast-mould heterogeneous domain using a weighted algorithm based on the homotopy perturbation method. *International Journal of Numerical Methods for Heat and Fluid Flow*.

[22] Nadeem M., He J. H. (2021). He–Laplace variational iteration method for solving the nonlinear equations arising in chemical kinetics and population dynamics. *Journal of Mathematical Chemistry*.

[23] Nadeem M., Yao S. W. (2021). Solving the fractional heat-like and wave-like equations with variable coefficients utilizing the Laplace homotopy method. *International Journal of Numerical Methods for Heat and Fluid Flow*.

[24] Habib S., Islam A., Batool A., Sohail M. U., Nadeem M. (2021). Numerical solutions of the fractal foam drainage equation. *GEM-International Journal on Geomathematics*.

[25] Wang K. (2022). A novel perspective to the local fractional Zakharov–Kuznetsov modified equal width dynamical model on cantor sets. *Mathematical Methods in the Applied Sciences*.

[26] Attia N., Akgül A., Seba D., Nour A., Riaz M. B. (2022). Reproducing kernel Hilbert space method for solving fractal fractional differential equations. *Results in Physics*.

[27] Zhang H., Nadeem M., Rauf A., Hui Z. G. (2021). A novel approach for the analytical solution of nonlinear time-fractional differential equations. *International Journal of Numerical Methods for Heat & Fluid Flow*.

[28] Yang X. J. (2016). A new integral transform method for solving steady heat-transfer problem. *Thermal Science*.

[29] Alesemi M., Iqbal N., Abdo M. S. (2022). Novel investigation of fractional-order Cauchy-reaction diffusion equation involving Caputo-Fabrizio operator. *Journal of Function Spaces*.

[30] Grzymkowski R., Hetmaniok E., Słota D. (2010). Application of the homotopy perturbation method for calculation of the temperature distribution in the cast-mould heterogeneous domain. *Journal of Achievements of Materials and Manufacturing Engineering*.

